# Matching Model of Dance Movements and Music Rhythm Features Using Human Posture Estimation

**DOI:** 10.1155/2022/7331210

**Published:** 2022-07-13

**Authors:** Dandan Jiang

**Affiliations:** Yangtze University, Jingzhou 434020, China

## Abstract

The essential issue in music understanding and dance synthesis research is how to improve the degree of matching between dance motions and music rhythm elements. The matching model of dance movements and music rhythm features is created in this study based on human posture estimation research to tackle the problems that existing matching methods are prone to rapid changes in movements and cannot keep the original movement features. The rhythm properties of movement and music data are first analyzed, and then the degree of matching between movement and music pieces is measured using a dynamic time warping technique. A constraint-based dynamic planning approach is also used to synthesize the dance action sequence that best matches the supplied music. Experiments reveal that this model has a matching accuracy of 95.1 percent, which is higher than the two comparative models' matching accuracy of 5.2 percent and 7.6 percent, respectively. The matching score of this paper is high, reaching around 94 percent, according to the user research results. The method suggested in this work has apparent advantages in that it may efficiently help users in the arrangement of desired dance moves or backing music, and it can be applied in the field of actual choreography and scoring.

## 1. Introduction

Music, as we all know, has the power to inspire people and to express themselves in various ways. “Rhythm” [1] is the element of music that has absolute appeal to individuals. The duration of music and the intensity of timbre make up rhythm [2]. The length relationship between the action and the time value in the process of completing the dance action is referred to as dance rhythm. Long, short, strong, and weak, and their relationships create dance movements' regularity through alternation, repetition, change, and contrast [3]. You may communicate the rhythm, melody, mode, and emotion of music through dance. Human beings' evolved artistic expression is dance with music. When listening to music, many people may unconsciously dance [4]. Professional dancers will carefully control their dancing with the music based on their previous expertise, in order to more accurately represent the feelings expressed in the song. The emotions portrayed by music in dance might be playful and attractive, gorgeous and elegant, joyous and vibrant, or vigorous and unrestrained, all of which have specific dancing qualities. At the same time, the dancer's mastery of “rhythm” is reflected in his or her sense of rhythm. The dancers' perception and presentation of dance are directly affected by the rhythm. Professional dancers will tightly manage their dancing during a stage performance according to the melody, pace, and intensity of the music, in order to more accurately portray musical feelings through dance. Professional choreographers frequently create tight rules for the synchronization of dance and music. Choreography is a difficult and talented job that requires this type of dance design effort.

Although a skilled dancer can match music and dance movements manually, it takes a lot of time. And compared with the editor of solo dance, everyone's posture in group dance is different, and the editing work will be more complicated. Therefore, it is of practical value to make the computer match the characteristics of dance movements and music rhythm, and its intelligence and automation are of certain practical value to dance arrangement. Action and music are time-series signals of two different perceptual channels. In order to properly evaluate the matching degree between them, it is necessary to establish a reasonable matching model between dance action and music rhythm. Human pose estimation is the basis of many tasks in the computer vision field [5–7]. It involves many disciplines, such as pattern recognition, image processing, computer vision, and artificial intelligence. It can be used in human-computer interaction, motion analysis, motion recognition, and other fields [8, 9]. At present, in the field of human posture estimation, convolutional neural network, as a representative algorithm of deep learning, has the ability of representation learning. Compared with traditional computer vision technology and expert system, it has better performance in target detection and recognition, natural language processing, and other fields. Therefore, this paper applies convolutional neural network to human posture estimation and constructs a matching model between dance movements and music rhythm features based on human posture estimation. Its innovations are as follows:

1. Based on the motion capture data, this paper constructs a motion database to store the rhythm and intensity characteristics of each motion segment. And in order to synthesize the dance action sequence that best matches the input music, a constraint-based dynamic planning process is introduced. Thereby, improving the matching degree of music and dance features and the smoothness of the resulting action sequence.
2. The pyramid pool layer is utilized at the end of the feature extraction module to consider the features of multilayer convolution more thoroughly. The attention network based on time dimension features is added after the pooling layer, the relevance weight is added to the features in the video frame, and the weight of the features is updated through iteration of the attention mechanism. Simultaneously, the upgraded 3D network is trained on the input data using various combinations of diverse data, and the best input data format is chosen by assessing the trial outcomes of various groups. Experiments suggest that this strategy can significantly increase the network's accuracy.

## 2. Related Work

In modern music, the matching of dance movements and musical rhythm features has been widely used in choreography and score, and the practical value of all aspects and the complexity of technology have become a problem worthy of further study. Many scholars have studied the feature analysis and feature matching of dance and music. The research contents and emphases are also different.

Romina et al. first extracted musical features such as rhythm, beat position, and dynamic features, and then controlled the actions of character animations according to predefined feature mapping criteria. This method can realize the synchronization of music and dance movements, but due to the limitation of mapping criteria, the generated dance movements are relatively monotonous, and cannot reflect the intrinsic connection between music and dance [10]. Nabila et al. took the different movement rhythms and bouncing techniques of dance as the research objects, and took the students of a dance art school as the experimental objects; from the various processing methods of the action rhythm, they showed different bouncing techniques, showing different dances or dance styles, and the matching relationship between dance and music was studied [11]. Vincent et al. used machine learning to construct the mapping relationship between movements and music from a database of samples and proposed a method to create dance movements based on the emotion and content of the music [12]. Jola et al. took the rhythm pattern of the movement as the main feature of the movement and combined the speed curves of the hands, feet, and center of gravity of the body when analyzing the rhythm of traditional dance [13]. Yu et al. proposed a rhythmic feature-based action-music matching model. However, the model ignores other features than rhythm, and the generated dance movements need to be improved in terms of globality and coordination [14]. Zhang et al. propose a rhythm analysis method. In this method, the extreme point of joint angular velocity is taken as the candidate point of the segmentation rhythm, and then it is refitted into the action characteristic curve according to the distribution of the candidate points [15]. In terms of music feature analysis, Xue et al. comprehensively analyzed the rhythm of music with features such as note onset, chord change, and drum pattern and used information such as music playback speed and tempo as the main music features [16]. In order to synthesize dance movements, Zhu et al. first analyzed the music and extracted the music beats, and then, based on the original movement database, they used the movement generation method to generate new movement data. The method for music and dance synthesis is based on the beat of the music, ignoring other musical features [17]. Burnett et al. believe that dance is an orderly organization of basic movements according to a certain theme. And by setting several basic movements and scheduling rules to generate music-independent dance sequences, and then editing the dance appropriately when it matches the music [18]. Govindan et al. proposed a method to synthesize music and dance synchronously according to the rhythm and intensity characteristics of movements and music. The main idea is that musical rhythm is strongly correlated with action rhythm, and the musical intensity that represents musical mode is also strongly correlated to the action intensity that represents action strength [19]. Mir et al. proposed a genetic algorithm to match rhythms. The genetic algorithm modifies the movements based on the generated movements to improve dance diversity. This method searches for candidate actions by constructing action graphs in advance, which improves the search efficiency of the choreography system. However, this method only utilizes rhythm matching and does not fully exploit other relevant features of actions and music [20].

This paper makes an in-depth study of related literature, summarizes the shortcomings and advantages, and constructs a matching model of dance movements and music rhythm features based on human posture estimation. Firstly, the underlying features of music and action are extracted, and some feature pairs are excluded by correlation analysis. Then, genetic algorithm is used to optimize and select the corresponding relationship between matching accuracy and operation speed. At the same time, in order to obtain the mapping relationship between movements and music, we train the sample data and get the evaluation function of the matching degree between dance and music. Based on the rhythm and intensity, the feature matching analysis of music segments and action segments is carried out, and according to the rhythm matching, the most matched action segments are screened out for each music segment. Then, connectivity analysis is carried out on adjacent action segments, and a plurality of result action sequences are obtained according to the connectivity, and then the most matched action sequence is obtained according to intensity matching. Finally, the experimental comparison with other different models shows that the performance of this model is better. This method is feasible and practical.

## 3. Methodology

### 3.1. Analysis and Extraction of Rhythm Characteristics of Dance and Music

It is a common feature of rhythm, dance, and music. First, select a set of optimal motion and music features, which should be able to reveal the features of motion and music data most effectively, thus facilitating the analysis of the relationship between music and motion. In order to fully tap the local correlation between music and dance and improve the richness of generated dance, this paper does not match the input music directly with the actions in the action database. Instead, the target audio is segmented first, and then feature matching is performed for each music segment and action segment. Therefore, the music needs to be segmented. The average length of the movements and music pieces used in this paper is about 2 seconds. Cutting the data into action segments can not only fully mine the features in finer granularity but also greatly facilitate the reuse of action data.

Assuming that the overall music sequence is denoted as *M*, after the music is segmented, *m* music segments are obtained, and denoted as

(1) $$\begin{array}{c} M_{1},M_{2},\ldots ,M_{m},\\ M=\left[M_{1},M_{2},\ldots ,M_{m}\right]. \end{array}$$

The extraction of music features is all based on music segments, and the music segments *M*_*i*_(1 ≤ *i* ≤ *m*) mentioned later all refer to the music segments in the music sequence *M*. The music features extracted by the music fragment *M*_*i*_ are recorded as

(2) $$\begin{array}{c} \text{Music }Feature\left(f\right)=\left[\begin{array}{c} F_{R}^{\text{Music}}\left(f\right)\\ F_{I}^{\text{Music}}\left(f\right) \end{array}\right]\;f\in M_{i}. \end{array}$$

Among them, *f* is the frame number of the music segment *M*_*i*_, and *F*_*R*_^Music^ and *F*_*I*_^Music^ are the rhythm and intensity features of the music segment, respectively.

For the vast majority of music segments, the quarter-note position of a music bar is often the starting point of all kinds of notes, and it is also the stress of the music, so the quarter-note position often coincides with the beat position of the notes. Music spectrum analysis provides the basis for music segmentation, music rhythm extraction, and music intensity extraction. Since the feature matching of music and action is based on the common features of music and action, namely rhythm and intensity, it is necessary to extract the rhythm and intensity features of music. In this paper, we adopt the following eight basic audio features: amplitude envelope, spectrum, cepstrum, spectrum histogram, periodicity histogram, fluency pattern, root-mean-square energy, and low-energy rate. The original music signal is a waveform signal in the time domain, but in order to extract richer information of music, such as rhythm and intensity, it is necessary to transform the music signal from the time domain to frequency domain and then analyze it. In order to ensure the stability of music rhythm and match with the internal structure of action bars, this paper only selects 4/4 beats of music pieces, and the music sequence is divided into music nodes according to bars. The map and workflow of this model are shown in Figure 1.

The mannequin used in this paper is a skeleton structure of human body, and the skeleton is composed of joint points that make up the human body. Human joints include head, hip, shoulder, chest, upper limbs, and lower limbs. These joint points constitute the human skeleton model according to the hierarchical relationship, with the hip as the root node, and other joint points are represented by rotation and displacement relative to their parent nodes. The orientation change of the rotation sub-joint point relative to the joint point is defined, and the displacement represents the spatial distance between the joint point and the sub-node. Each of the correlation coefficients may be the clue of the mapping relationship between action and music. However, considering all the coefficients at the same time will bring a very heavy amount of calculation. And some coefficient components will bring noise to the correlation between mining action and music. Therefore, this paper adopts the optimal feature selection algorithm to extract a representative feature subset, which should effectively represent the relationship between action-music and reduce unnecessary noise. Since the feature matching of music and action is based on the common features of music and action and rhythm and intensity, it is necessary to extract the rhythm and intensity features of action. In order to fully mine features in finer granularity and facilitate the reuse of action data, actions are segmented. The action mode is the same as the music segmentation mode above.

The action speed m_velocity of the joint point refers to the displacement of the joint point of the human body in unit time, and its calculation method is as follows:

(3) $$\begin{array}{c} m\_velocity=\frac{f_{i}\left(j+1\right)-f_{i}\left(j\right)}{\Delta t}, \end{array}$$

wherein, *f*_*i*_(*j*) represents the position of the joint point *i* at the *j*th frame; *f*_*i*_(*j*+1) − *f*_*i*_(*j*) represents the position change of the joint point *i* at the frame *j*; Δ*t* is the time length of the *j*th frame. The formula for calculating the acceleration of the action is as follows:

(4) $$\begin{array}{c} m\_acceleration=\frac{v_{i}\left(j+1\right)-v_{i}\left(j\right)}{\Delta t}. \end{array}$$

Among them, *v*_*i*_(*j*) represents the velocity of the joint point *i* at the *j*th frame. The formula for calculating the action distance is as follows:

(5) $$\begin{array}{c} C_{i}=\frac{1}{N}\left(\sum_{j=1}^{N}f_{i}\left(j\right)\right),\\ m\_\text{span}=\sum_{i=2}^{n}\sum_{j=1}^{N}\left|f_{i}\left(j\right)-C_{i}\right|. \end{array}$$

Among them, *C*_*i*_ is the center position of all positions of the ith joint point of the human body in the action clip, *N* represents the number of frames in the action clip, and n represents the number of joint points used in the human body model.

Because every joint point of an action segment can construct a cosine curve, in order to fully express the characteristics of the whole action, it is necessary to compound the curves of specific joint points that users are interested in, and the compound curve obtained by weighted average of each curve is the whole action curve. Static features are used to describe the pose characteristics of human characters. The static features extracted in this paper include motion spacing, motion density, arm shape, foot footprint, and balance. Traditional rhythm extraction methods that only aim at certain types of dance movements have great limitations. Because the feature extraction of the motion data is preprocessed and stored in the motion database, it can be extracted manually by its suitable rhythm extraction algorithm according to the dance style.

### 3.2. Construction of the Match Model between Motion and Music Features

Human pose estimation can be simply regarded as the combination of feature extraction [21] and classifier recognition. From preprocessing to feature selection, human motion information is extracted from the underlying data, and then classified by classifier to complete motion recognition. The process of human body motion recognition is the process of acquiring high-level motion information through the underlying data, thus learning the motion characteristics and finally realizing the motion classification. When estimating the human posture, the input data are the video frame sequence, so we need to consider not only the spatial representation of actions but also the sequence of atomic actions in the video frame sequence. There are three types of motion feature extraction based on nondeep learning algorithm: low-level features, middle-level, and high-level features and silhouettes. Low-level features usually refer to spatio-temporal interest points and dense optical flow. And middle-level features, mainly long-term tracking track or semantic representation. The premise of recognizing human movements by silhouette features is to assume that human movements are regarded as a continuous process of body posture. The learning process is extracted from a series of silhouettes, and then the traditional classifier is used to identify human movements. According to different application requirements, some researchers use single-view data, but the results are often vague. Especially in the method based on target silhouette, the system falls into local minima because multiple poses correspond to the same silhouette. Moreover, the traditional 2D convolution network cannot deal with the sequence of atomic actions when dealing with motion recognition in video, which has great limitations. This problem can be solved in 3D convolution network.

Assuming that the neuron has three input values: *x*_1_, *x*_2_, *x*_3_, and the output is as follows:

(6) $$\begin{array}{c} h_{W,b}\left(x\right)=f\left(\sum_{i=1}^{3}W_{i}x_{i}+b\right), \end{array}$$

where *W*_*i*_ and b are the neuron parameters at the input and *f*(·) is the activation function. Sigmoid function

(7) $$\begin{array}{c} \sigma \left(x\right)=\frac{1}{1+\exp\left(-x\right)}. \end{array}$$

Hyperbolic tangent tanh function

(8) $$\begin{array}{c} \tanh\left(x\right)=\frac{e^{x}-e^{-x}}{e^{x}+e^{-x}}. \end{array}$$

The rhythm of the dance is synchronized with the music. Dancers always step on the rhythm points of the music when dancing, similar to clapping and beating, which can be roughly regarded as the coincidence of the stop action and rhythm points of the dancers. For each action and music segment combination, we extract 40 music features and 455 action features. Through correlation analysis, a correlation coefficient can be obtained, which together form a correlation coefficient matrix. Theoretically, the rate of change of eigenvalues can better reflect the development and change of things than the eigenvalues themselves. For a given well-matched action and music piece, the greater the change of the action part, the worse the matching degree with the original music piece. Feature matching is mainly based on rhythm and intensity matching. However, in order to ensure that the action segments can finally be connected into a coherent and natural dance action, it is necessary to analyze the connectability between every two adjacent action segments whose rhythm matches each music segment. In this chapter, the connectability analysis controls the current action and the previous action. When the adjacent action is the same action, the action distance between them is set to infinity, so that when the adjacent action is the same action, the two actions cannot be connected. The algorithm flow is shown in Figure 2.

In order to obtain positive training samples, all matching action-music piece combinations can be selected as positive training samples. We randomly chose a clip from all captured action footage and coupled it with a music clip to collect examples of negative training. The algorithm is used to determine the combination's matching score for each action-music piece combination. We can discover the best matching K music nodes for each action segment by comparing the scores, and these matching results will then be placed in an action-music mapping table. Similarly, a tag is provided for rhythm matching of dance action database with strong rhythm for music.

Let {*v*_*i*1_, *v*_*i*2_,…, *v*_*iK*_} and {*v*_*j*1_, *v*_*j*2_,…, *v*_*jK*_} be the set of *K* music nodes that best match *u*_*i*_ and *u*_*j*_ obtained from the map, respectively. Then, the music edges corresponding to *u*_*i*_ and *u*_*j*_ are the directed edges *v*_*im*0_ and *v*_*jn*0_ with the smallest distance in the music graph in

(9) $$\begin{array}{c} v_{im0}\in \left\{v_{i1},v_{i2},\ldots ,v_{iK}\right\},\\ v_{jn0}\in \left\{v_{j1},v_{j2},\ldots ,v_{jK}\right\}. \end{array}$$

Therefore, the music nodes *v*_*im*0_ and *v*_*jn*0_ can be used as the background music corresponding to the action nodes *u*_*i*_ and *u*_*j*_, respectively. The corresponding dance moves are calculated in the same way. The matching error of the action and the music is estimated as follows:

(10) $$\begin{array}{c} L\left(A_{j},M_{j}\right)\overset{\Delta }{=}1-\exp\left(-{\text{Dist}}_{m}\left(M_{i},M_{j}\right)\right). \end{array}$$

In this paper, we choose a specific correlation coefficient for each dance. The termination condition of feature coefficient selection is that when six new correlation coefficients are allowed to be selected into this subset, the accuracy should be increased by at least 4%. Start with an empty feature subset and add new features to the set until the termination condition is not met. The size setting of threshold is a measure of cohesion and connectivity. If the threshold setting is small, the adjacent actions are very similar, and the cohesion is very coherent, but the connectible action sequences will decrease accordingly. Anyway, if the threshold setting is large, the adjacent actions will be connected without being very similar, resulting in poor connection, but the connectible action sequence will increase accordingly. In addition, threshold setting has different requirements for different action types. Music-action correspondence is a set of music-action feature pairs, which is used for the matching calculation of music and dance. The music features and action features that make up the feature pair are in one-to-one correspondence and have high correlation characteristics.

In order to extract connectible actions based on connectivity, this section proposes a graph-based depth-first traversal algorithm for extracting connectible actions. Each action segment is regarded as a node, and a directed edge is established according to whether adjacent segments are connected or not. If adjacent segments are connectible, a directed edge is established; On the other hand, if the adjacent segments are not connectible, there is no directed edge in the adjacent segments. According to the best matching path of the sequence of motion and music feature points given by this algorithm, the motion (music) segment can be deformed to map the motion (music) feature points to the corresponding music (motion) feature points, thus further improving the matching degree between the motion and music segments.

## 4. Result Analysis and Discussion

The algorithm proposed in this paper is tested on multiple sequences, including synthetic and real data. The configuration of the experimental platform is Intel Pentium D2.80 GHz CPU, 16 GB memory, and uses QT4.2 and MatLab development environment. Dance sequences were acquired at a frame rate of 30 fps using a motion analysis optical motion capture device. The size of the voxels in the experiment is set to 18 × 18 × 18. The dance movements used are recorded as movement data in BVH format. The data have 65 degrees of freedom, which contain 24 joint points, each joint point has about 2 degrees of freedom. The actions are recorded to the file at a frame rate of 35 frames per second. The accompanying background music is all single-channel music with a sampling frequency of 45 kHz. The sampling rate of the motion data is 35 Hz. The music in WAV audio format is extracted from the video file by the software Adobe Premiere, and the parts without sound at the beginning and end of the video are manually removed. In the experiment, an action graph containing 1069 nodes is constructed, and each node corresponds to an action segment. The total node length is about 726 seconds. The comparison results of the corresponding relationship accuracy of the underlying features and the corresponding relationship accuracy of the high-level statistical features are shown in Table 1.

From the experimental data in Table 1, it can be seen that, compared with the high-level statistical features, using the low-level features to construct the music-action correspondence can get higher accuracy. While the accuracy of the correspondence of high-level statistical feature is relatively low. In order to test the rationality of matching the characteristics of music rhythm and intensity with those of dance movements, several experiments were designed. In order to evaluate the effectiveness of the method proposed in this paper, the F1 index, which can comprehensively reflect the performance of the algorithm is selected to experiment the algorithm in this paper and compare different algorithms, and the result shown in Figure 3.

In practical application, the action map and music map in the action-music map are mostly composed of the same kind of dance, so the matching quality of the result animation created by the system when the action map and music map are constructed by the same kind of dance is evaluated. Every time it is necessary to determine an action segment from the candidate action set, the action segment with the best coherence is the first. Then randomly choose one of them as the action segment of the matching music. All initial postures are chosen from the live dance of motion capture. From the existing music-action database, based on the music similarity and the input music, the music-action data with corresponding matching are obtained, and the path of its action data is extracted as the reference path. When the action map part and music map part of the action-music map are composed of different dance types, the difference of style between the action bar and the music bar may lead to the change of algorithm performance. This paper also evaluates the matching quality for this situation. The accuracy of matching dance movements with music rhythm features by different methods is shown in Figure 4.

The matching action sequences can be counted, and if a certain number of values are reached, the traversal can be terminated. Because every time an adjacent point is visited, the adjacent point with the best rhythm is preferentially visited, so the action sequence obtained in priority matches the rhythm of the input music signal better. This paper puts forward the definition of fluency function and uses quantitative data to objectively analyze the connection between dance movements and music matching. The cohesion of dance movements using different matching methods is shown in Figure 5.

It can be seen that the dance movement cohesion of this matching method is obviously higher than that of the other two methods.  Table 2 shows the time performance evaluation in this chapter. In this test, the time performance differences of the method in reference [11] and the method in reference [17] are compared.

In the methods of literature [11] and literature [17], it is important to traverse the music or action graph for each action or music segment to locate the best matching music node. We simply need to query the map for the best matched node in our function. As a result, our method's search speed is substantially faster than the other two techniques. 150 students were asked to complete a user experience research in order to objectively evaluate and test the model's performance. A user ability test was conducted prior to the experiment to guarantee that the participants could actually identify whether the action matched the music. Experimenters who did not have a strong musical background or who had difficulty appropriately perceiving the movement-music connection were removed. The user research study drew a total of 100 participants.  Figure 6 depicts the pleasure of these 100 students with various model matching results.

In order to give more credibility to the evaluation results, we will compare the degree of difference between human and machine ratings. The results of automatic scoring by the algorithm are shown in Figure 7.

From the comprehensive analysis of the data in the two figures, it can be seen that the result of manual scoring is very similar to that of algorithm scoring. This also verifies the reliability of the score and draws the conclusion that the dance movements of this paper match the rhythm features of music to a high degree. According to the experiments in this chapter, the matching accuracy of this model is as high as 95.1%, which is higher than 5.2% and 7.6% of the two comparative models, respectively. This model effectively improves the efficiency and accuracy of the choreography and score system. And the matching score of this paper is high, reaching about 94%. It can be used in the field of actual choreography and score.

## 5. Conclusions

This is the law according to which rhythmic sequence and movements develop. Based on the estimation of human posture, this paper constructs a feature matching model of dance movements and music rhythm, which solves the problem of matching movements and music well. Firstly, based on the synchronization number of rhythm points of music and dance movements in time, the paper carries out rhythm matching. And in order to ensure the cohesion of adjacent action segments, the connectability analysis of adjacent action segments is made based on the action distance. At the same time, in order to generate the optimal dance action sequence, a dynamic planning process based on constraints is introduced. This process takes into account both the matching degree between actions and music and the coherence degree between actions in the result. The experimental results show that the matching score of this paper is high, reaching about 94%. And the matching accuracy of this model is as high as 95.1%, which is higher than 5.2% and 7.6% of the two comparative models, respectively. From the database point of view, this model effectively improves the efficiency and accuracy of the choreography and score system. The integration of movement and music has always been a difficult problem, which needs to be improved and dealt with at a deeper level. Although some research achievements have been made in this paper, the score algorithm of this paper has not considered enough the harmony of the transition between music pieces, and this content will be studied in depth in the next step.

## Figures and Tables

**Figure 1:** Workflow of the model in this paper.

**Figure 2:** Algorithm flow.

**Figure 3:** F1 value comparison.

**Figure 4:** Matching accuracy of different methods.

**Figure 5:** Dance movement cohesion results of different matching methods.

**Figure 6:** Satisfaction comparison of matching results of different models.

**Figure 7:** The result of the automatic scoring of the algorithm.

**Table 1:** Comparison of the accuracy of the corresponding relationship between low-level features and high-level statistical features.

Music number	Low-level feature correspondence accuracy	High-level statistical feature correspondence accuracy		
		SHI	KIM	SMS
1	77.6	67.2	70.9	69.8
2	75.4	60.3	67.5	71.4
3	76.3	64.7	65.9	72.3
4	74.5	71.3	70.5	69.4
5	76.8	68.4	69.7	62.8

**Table 2:** Time efficiency comparison of choreography and soundtrack of different systems.

Choreographer	Soundtrack								
Serial number	Number of feature points	Literature [11] method	Literature [17] method	Method of this paper	Serial number	Number of feature points	Literature [11] method	Literature [17] method	Method of this paper
1	30	44.69	43.14	16.24	5	25	30.98	31.46	13.27
2	32	46.59	45.87	17.58	6	20	25.87	24.96	11.54
3	35	50.16	50.34	19.24	7	23	28.49	27.68	12.63
4	37	53.19	52.87	21.16	8	19	20.39	21.58	10.01

## Data Availability

The data used to support the findings of this study are available from the corresponding author upon request.
